# Occurrence of the Foramen of Vesalius and Its Morphometry Relevant to Clinical Consideration

**DOI:** 10.1100/2012/817454

**Published:** 2012-05-02

**Authors:** Vipavadee Chaisuksunt, Lanaprai Kwathai, Kritsana Namonta, Thanaporn Rungruang, Wandee Apinhasmit, Supin Chompoopong

**Affiliations:** ^1^Department of Anatomy, Faculty of Medicine, Chiang Mai University, Chiang Mai 50200, Thailand; ^2^Department of Anatomy, Faculty of Medicine Siriraj Hospital, Mahidol University, Bangkok 10700, Thailand; ^3^Department of Anatomy, Faculty of Dentistry, Chulalongkorn University, Bangkok 10330, Thailand

## Abstract

All 377 dry skulls were examined for the occurrence and morphometry of the foramen of Vesalius (FV) both in the middle cranial fossa and at the extracranial view of the skull base. There were 25.9% and 10.9% of FV found at the extracranial view of the skull base and in the middle cranial fossa, respectively. Total patent FV were 16.1% (11.9% unilaterally and 4.2% bilaterally). Most FV were found in male and on the left side. Comparatively, FV at the extracranial view of the skull base had a larger maximum diameter. The distance between FV and the foramen ovale (FO) was as short as 2.05 ± 1.09 mm measured at the extracranial view of the skull base. In conclusion, although the existence of FV is inconstant, its occurrence could not be negligible. The proximity of FV to FO should remind neurosurgeons to be cautious when performing the surgical approach through FO.

## 1. Introduction

Among several foramina on the greater wing of sphenoid bone, the inconstant foramen of Vesalius (FV) connects the pterygoid plexus with the cavernous sinus and transmits a small emissary vein which drains the cavernous sinus [1]. The importance of this foramen is that it offers a path to the spread of an infection from the extracranial source to the cavernous sinus. The small FV, if present, is generally situated posteromedially from the foramen rotundum (FR) and anteromedially from the foramen ovale (FO), foramen spinosum (FS), and carotid canal [2]. The FV is located between the FO and FR, but particularly more closely to the FO, and thus neurosurgery may misplace the needle during percutaneous intervention targeting the FO for treatment of the trigeminal neuralgia, resulting in severe complications such as intracranial bleeding [3]. However, this foramen is considered as an inconstant channel and has a widely variation reported by several studies [2–6]. Therefore, the present study aimed to evaluate the frequency of occurrence and the morphometry of the FV in Thais, and these anatomical considerations may assist the surgeon to a better planning and a safer execution of percutaneous approach to the middle cranial fossa through the FO.

## 2. Materials and Methods

The present study was designed as a descriptive study. The experimental protocols of this study have been approved by the Ethics Committee of two universities from which the skulls were selected, that is, Faculty of Medicine Siriraj Hospital, Mahidol University, and Faculty of Medicine, Chiang Mai University, Thailand.

Bilateral sides of 377 Thai adult dry skulls were selected from the collections at the Department of Anatomy of two universities, Faculty of Medicine Siriraj Hospital, Mahidol University, and Faculty of Medicine, Chiang Mai University. All skulls were known of their sex and age according to the personal records of body donors. Only skulls in regular shape, without obvious evidence of dystrophy, deformities, and/or trauma, were selected. Criteria of exclusion were those in which the partly surrounding bones of the FV were broken.

For the evaluation of occurrence of the FV, the skulls were directly examined for the presence of the FV separately in the middle cranial fossa and at the extracranial view of the skull base and recorded in designed data sheets if it was found. To prove the patent FV, a wire with the diameter of 0.2 mm was inserted through the FV from the extracranial view of skull base to the middle cranial fossa.

For the morphometry of the FV, its location and dimensions were analyzed by using computer image analysis. In any skulls, where the FV was present, a digital camera was used to capture the FV from both sides of the skull base. Then, Image Tool 3.0 Program (UTHSCSA, The University of Texas Health Science Center in San Antonio, USA) was used to measure the maximum and minimum diameters of the FV and the distance between the FO and FV. Because of the irregular shape of both foramina, the distances were measured from the nearest margin of each foramen to avoid overestimated values.

Each measurement was performed three times and averaged. All measurements and frequencies of the data were tabulated and separated according to sex, side, and symmetrical groups. Statistical Package for the Social Science (version 11.5) software (SPSS; Chicago, IL, USA) was used for the analysis. The Chi-square test was used to test for differences of the FV groups and the percentage values. The mean and standard deviation (SD) of measurements were assessed and expressed as Mean ± SD. The comparison of values between sexes was made using the unpaired *t*-test, whereas that between sides was made using the paired *t*-test. The level of significant difference was *P* < 0.05.

## 3. Results

Three hundred and seventy-seven skulls were examined in the present study which comprised 246 males (65.3%) and 131 females (34.7%) with the mean age of 61.27 ± 16.74 years (13 to 94 years). There was no significant age difference between males (61.62 ± 16.31 years) and females (60.63 ± 17.58 years) (*P* = 0.588).

In this study, the FV was observed in both middle cranial fossa (Figure 1(a)) and extracranial view of the skull base (Figure 1(b)). It was always an independent structure lying on the greater wing of the sphenoid bone and in the neighborhood of the FO. This foramen could be found bilaterally (Figure 1(c)). It was located posteromedially to the FR and anteromedially to the FO and FS (Figures 2(a) and 2(b), resp.).

The present study was conducted in a total of 754 sides of 377 adult dry skulls (492 males and 262 females). The presence of the FV was calculated as a percentage of total sides of skulls as shown in Table 1. In both middle cranial fossa and extracranial view of the skull base, the FV was present in 10.9% (82 of 754 sides) and 25.9% (195 of 754 sides) of total sides observed, respectively. It was found more frequently in the extracranial view of the skull base than in the middle cranial fossa, on the left side more than on the right side, and in male more than in female (Table 1). Pearson Chi-square test indicated the significant difference of the frequency of FV only between in the extracranial view of the skull base and in the middle cranial fossa (*P* < 0.05). The absence of this foramen was found up to 89.1% (672 of 754 sides) in the middle cranial fossa and 74.1% (559 of 754 sides) at the extracranial view of the skull base.

When comparing the percentage of the FV found in total skulls as shown in Table 2, it was found more commonly at the extracranial view of the skull base (37.6%) than in the middle cranial fossa (17.2%). The FV was found unilaterally both in the middle cranial fossa (12.7%) and the extracranial view of the skull base (23.6%) more often than when it appeared bilaterally on either surface of the skull base (4.5% and 14.0%, resp.). In the middle cranial fossa, in a total of 82 sides of the skulls observed, the FV was present unilaterally in 48 sides of 48 skulls (16 right, 32 left) and bilaterally in 34 sides of 17 skulls (17 right, 17 left). Therefore, 17.2% of the FV were 12.7% unilateral FV (48 of 377 skulls) and 4.5% bilateral FV (17 of 377 skulls). At the extracranial view of the skull base, in a total of the 195 sides in which the FV was observed, the unilateral FV was found in 89 sides of 89 skulls (35 right, 54 left), and the bilateral FV was found in 106 sides of 53 skulls (53 right, 53 left). Therefore, 37.6% of the FV were 23.6% unilateral FV (89 of 377 skulls) and 14.0% bilateral FV (53 of 377 skulls).

Regarding sex, the percentage of skulls in which at least one foramen was found either in the middle cranial fossa or at the extracranial view of the skull base were higher in males (8.7% and 14.3%, resp.) than in females (4.0% and 9.3%, resp.) (Table 2). However, when inserting a wire through the FV from the extracranial view of the skull base to the middle cranial fossa to identify the patent FV, the result showed that the percentage of the patent FV was only 16.1%, of which 11.9% were the unilateral FV (45 of 377 skulls) and 4.2% were the bilateral FV (16 of 377 skulls) (Table 2).

The FV is a very small foramen with average diameters of 1.48 ± 0.65 mm in the middle cranial fossa and 1.70 ± 0.63 mm at the extracranial view of the skull base. The maximum diameter of the FV found at the extracranial view of skull base was larger significantly on the left side (2.58 ± 1.03 mm) than on the right side (2.29 ± 0.97 mm) (*P* < 0.05), but there was no significant difference related to sex (Table 3). In addition, the average distance between the FO and the FV at the extracranial view of the skull base (2.05 ± 1.09 mm) was shorter than that in the middle cranial fossa (2.78 ± 1.46 mm) significantly, and the same results were found when comparing between sexes and sides (*P* < 0.05).

## 4. Discussion

The FV is originally found as the emissary foramen by Andreas Vesalius [15]. At the base of skull, this foramen is located in the greater wing of the sphenoid bone and communicates between the extracranial and intracranial structures. Therefore, this study investigated the occurrence of the FV both in the middle cranial fossa and the extracranial view of the skull base. In addition, the real communication between the FV at extracranial and intracranial views of the skull base was proved by inserting wires and found that the percentage of the patent FV was only 16.1% of total skulls and that was less than the FV found in the middle cranial fossa (17.2%) and extracranial view of the skull base (37.6%). This result showed that most of the FV at the extracranial view of the skull base were blind channels.

Various studies have reported the occurrence of the FV and its variations [2–6]. In the present study, an occurrence of the FV was different from previous studies; in those studies, either higher or lower percentage of the presence of the FV was reported, for example, 100% in 10 skulls found by Kaplan et al. [8], 40% by Rossi et al. [5], 36.5% by Boyd [9], 33.8% in 400 skulls by Shinohara et al. [6], 32.9% by Gupta et al. [3], 22.0% by Reymond et al. [4], 21.8% by Kodama et al. [2], and 8.5% by William et al. [10]. According to Wysocki et al. [11], the FV could be found in 17.0% of 100 skulls. This occurrence is relatively similar to the finding of the present study (patent FV, 16.1% of 377 skulls).

The presence of the unilateral patent FV was 11.9% in this study, which is close to 13.0% in the study of Bergman et al. [12]. According to the previous reports, the frequency of the unilateral patent FV might be as high as 80% in the study by Ginsberg et al. [13], 26.5% by Rossi et al. [5], 20.0% by Gupta et al. [3], and 18.3% by Shinohara et al. [6] and as low as 5.5% by Kodama et al. [2]. Furthermore, the occurrence of the bilateral patent FV of 4.2% in this study was slightly lower than that of 5.0% reported by Reymond et al. [4] while it was much lower when compared to the occurrence of 35% reported by Berge and Bergman [14], 22% by Kodama et al. [2] and Gupta et al. [3], 15.5% by Shinohara et al. [6] 13.8% by Rossi et al. [5], and 12.5% by Boyd [9]. In addition, Kodoma et al. [2] and Gupta et al. [3] reported that the occurrence of the bilateral FV was greater than the unilateral FV, but in our study, like the observation by Ginsberg et al. [13], the unilateral FV was found more frequently than the bilateral FV. Interestingly, it was reported in the famous book by Vesalius [15] that there was no significant difference between the unilateral FV on the right and left sides of the skulls. Based on our results and other previous studies, the occurrence of the unilateral FV was found more commonly on the left side than on the right side [6, 9].

In this study, the maximum diameter of FV at the extracranial view of the skull base (2.45 ± 1.01 mm) was significantly larger than that in the middle cranial fossa (2.00 ± 0.91 mm) (*P* < 0.05). It was also significantly larger on the left than on the right side (*P* < 0.05). The results were similar to Rossi et al. [5] whose study found that the mean diameter of FV was 1.59 ± 0.94 mm on the left side and 1.46 ± 1.04 mm on the right side. However, Shinohara et al. [6] found the shorter diameter of the FV, that is, 0.72 mm on the left side and 0.69 mm on the right side whereas the observed diameter was up to 1-2 mm as reported by Lanzieri et al. [16].

The FV was situated anteromedially to the FO at the mean distance of 2.05 ± 1.09 mm at the extracranial view of the skull base and 2.78 ± 1.46 mm in the middle cranial fossa. The distance between the FV and FO measured in the middle cranial fossa was significantly greater than that in the other side of the skull base both on the left side (2.53 ± 1.30 mm) and the right side (3.15 ± 1.64 mm). The study of Shinohara et al. [6] showed no significant difference in the average FV-FO distance between the left (2.59 mm) and the right sides (2.55 mm), and this was close to the result in the middle cranial fossa (2.78 ± 1.46 mm) obtained from this study. On the contrary, the study of Rossi et al. [5] showed that the FV-FO distance on the right side of the skull was less than that on the left side (1.85 ± 0.30 mm and 2.46 ± 0.31 mm, resp.).

Due to the importance of the FV and the occurrence of the patent FV found in this study, it could be implicated that the possibility of the infection spreading from the extracranial origin or infratemporal region into the middle cranial fossa is up to 16.1%. This could occur because the emissary vein passing through this foramen connects the venous system of the face, through the pterygoid venous plexus, to the cavernous sinus [4]. In addition, using certain neurosurgical techniques such as radiofrequency rhizotomy for the treatment of trigeminal neuralgia by approaching through the FO, in case of the presence of the FV, the neurosurgeon should be aware of the proximity of two foramina, which could be as close as 2.05 ± 1.09 mm. Strong evidences from several previous studies showed that the misplacing of the needle from the FO could penetrate the FV, make a puncture in the cavernous sinus [17], the cave of Meckel, and cause bleeding in the temporal lobe [6]. As observed in the present study, the greater the diameter of the FV, the less the distance between the FV and FO. Taken together, neurosurgeons should be aware of the presence of the FV as a possible cause of complications during clinical treatments. In addition, misunderstanding might occur during the radiography interpretation. Even though some of the FV were blind channels, the occurrence of the patent FV was considerable (up to 16.1% in this study).

## 5. Conclusion

Owing to being a small and inconstant foramen, the FV is not routinely in attention during surgery. The knowledge of the occurrence of the FV may assist the neurosurgeon to realize that the FV is located very close to the FO, particularly at the extracranial view of the skull base. Therefore, in case it exists, the approach through the FO could be the more complicated procedure and the operation should be carefully performed to avoid the FV puncture.

## Figures and Tables

**Figure 1:** The FV viewed from the middle cranial fossa (a) and the extracranial view of the skull base (b). Panel (c) shows an example of the bilateral FV in the extracranial view of the skull base. The asterisks (*) in (a) and (b) indicate a bony process which probably hinders the approach of the structures passing through the FO. CC: carotid canal; FL: foramen lacerum; FO: foramen ovale; FS: foramen spinosum; FV: foramen of Vesalius.

**Figure 2:** The patent FV viewed from the middle cranial fossa (a) and the extracranial view of the skull base (b). CC: carotid canal; CG: carotid groove; FL: foramen lacerum; FO: foramen ovale; FR: foramen rotundum; FS: foramen spinosum; FV: foramen of Vesalius.

**Table 1:** Distribution of the FV found in analyzed dry skulls according to side and sex.

Groups	*N* (sides)	FV [sides (%)]	
		Middle cranial fossa	Extracranial view of the skull base
Right side	377	33 (8.8)	88 (23.3)
Left side	377	49 (13.0)	107 (28.4)

Male	492	61 (12.4)	134 (27.2)
Female	262	21 (8.0)	61 (23.3)

Total sides	754	82 (10.9)	195 (25.9)

**Table 2:** Distribution of the unilateral and bilateral FV found in analyzed dry skulls according to side and sex.

Groups (*N*, skulls)	Patent FV [Skulls (%)]			FV in middle cranial fossa [Skulls (%)]			FV in extracranial view of the skull base [skulls (%)]		
	Right side	Left side	Total sides (*N* = 377)	Right side	Left side	Total sides (*N* = 377)	Right side	Left side	Total sides (*N* = 377)
Unilateral FV	14 (3.7)	31 (8.2)	45 (11.9)	16 (4.2)	32 (8.5)	48 (12.7)	35 (9.3)	54 (14.3)	89 (23.6)
Male (246)	10 (2.7)	21 (5.6)	31 (8.2)	12 (3.2)	21 (5.6)	33 (8.7)	20 (5.3)	34 (9.0)	54 (14.3)
Female (131)	4 (1.1)	10 (2.7)	14 (3.7)	4 (1.1)	11 (2.9)	15 (4.0)	15 (4.0)	20 (5.3)	35 (9.3)

Bilateral FV			16 (4.2)			17 (4.5)			53 (14.0)
Male (246)			13 (3.4)			14 (3.7)			40 (10.6)
Female (131)			3 (0.8)			3 (0.8)			13 (3.4)

**Table 3:** Comparison the diameters of FV and the distance between FV and FO according to sides and sexes.

Measurements (mm)	Total sides		Right side		Left side		Male		Female	
	*N*	Mean ± SD	*N*	Mean ± SD	*N*	Mean ± SD	*N*	Mean ± SD	*N*	Mean ± SD
FV in the middle cranial fossa										

Maximum diameter	40	2.00 ± 0.91^a^	17	1.71 ± 0.58	23	2.22 ± 1.05	29	2.10 ± 1.01	11	1.75 ± 0.54
Minimum diameter	40	0.96 ± 0.48	17	0.92 ± 0.47	23	0.98 ± 0.50	29	0.97 ± 0.53	11	0.91 ± 0.33
Average diameter	40	1.48 ± 0.65	17	1.31 ± 0.46	23	1.60 ± 0.74	29	1.53 ± 0.73	11	1.36 ± 0.33
FV-FO distance	39	2.78 ± 1.46^b^	16	3.15 ± 1.64	23	2.53 ± 1.30	29	2.67 ± 1.52	10	3.11 ± 1.27

FV at the extracranial view of the skull base										

Maximum diameter	200	2.45 ± 1.01^a^	90	2.29 ± 0.97^c^	110	2.58 ± 1.03^c^	136	2.45 ± 1.05	64	2.44 ± 0.93
Minimum diameter	200	0.96 ± 0.46	90	0.99 ± 0.44	110	0.93 ± 0.48	136	0.97 ± 0.48	64	0.93 ± 0.41
Average diameter	200	1.70 ± 0.63	90	1.64 ± 0.61	110	1.75 ± 0.64	136	1.71 ± 0.65	64	1.68 ± 0.57
FV-FO distance	201	2.05 ± 1.09^b^	90	2.05 ± 1.17	111	2.05 ± 1.03	136	2.06 ± 1.15	65	2.02 ± 0.97

^a–c^Significant difference between groups which are indicated with the same alphabet at *P*  value < 0.05.
